The article "Integrative Analyses of Biomarkers Associated with Endoplasmic Reticulum Stress in Ischemic Stroke" was published in 2022. Journal: Comput Math Methods Med.

# Integrative Analyses of Biomarkers Associated with Endoplasmic Reticulum Stress in Ischemic Stroke

**DOI:** 10.1155/2022/4212180

**Published:** 2022-08-25

**Authors:** Xiaoting Zhang, Xi Li, Jinyan Gu, Jingpei Guo, Jiayao Chen, Ke Zhang, Junfeng Liu, Jiani Liu, Chao Peng, Hanwei Liu, Bin Zhou

**Affiliations:** ^1^Center of Interventional Medicine, The Fifth Affiliated Hospital of Sun Yat-sen University, Zhuhai, Guangdong Province, 519000, China; ^2^Library, The Fifth Affiliated Hospital of Sun Yat-sen University, Zhuhai, Guangdong Province, 519000, China; ^3^Guangdong Provincial Key Laboratory of Biomedical Imaging and Guangdong Provincial Engineering Research Center of Molecular Imaging, The Fifth Affiliated Hospital of Sun Yat-sen University, Zhuhai, Guangdong Province, 519000, China

## Abstract

**Background:**

Neuronal apoptosis, which is the primary pathological transform of cerebral injury following ischemic stroke (IS), is considered to be induced by endoplasmic reticulum stress (ERS) by numerous reports. However, ERS biomarkers in IS have not been fully identified yet. Consequently, the present study is aimed at exploring potential blood biomarkers by investigating the molecular mechanisms of ERS promoting neuronal apoptosis following IS development.

**Methods:**

A comprehensive analysis was performed with two free-accessible whole-blood datasets (GSE16561 and GSE37587) from the Gene Expression Omnibus database. Genetic information from 107 IS and 24 healthy controls was employed to analyze the differentially expressed genes (DEGs). Genes related to ERS (ERS-DEGs) were identified from the analysis. Enrichment analyses were performed to explore the biofunction and correlated signal pathways of ERS-DEGs. Protein-protein interaction (PPI) network and immune correlation analyses were performed to identify the hub genes along with their correspondent expressions and functions, all of which contributed to incremental diagnostic values.

**Results:**

A total of 60 IS-related DEGs were identified, of which 27 genes were confirmed as ERS-DEGs. GO and KEGG enrichment analysis corroborated that upregulated ERS-DEGs were principally enriched in pathways related to immunity, including neutrophil activation and Th17 cell differentiation. Moreover, the GSEA and GSVA indicated that T cell-related signal pathways were the most considerably immune pathways for ERS-DEG enrichment. A total of 10 hub genes were filtered out via the PPI network analysis. Immune correlation analysis confirmed that the expression of hub genes is associated with immune cell infiltration.

**Conclusions:**

By integrating and analyzing the two gene expression data profiles, it can be inferred that ERS may be involved in the development of neuronal apoptosis following IS via immune homeostasis. The identified hub genes, which are associated with immune cell infiltration, may serve as potential biomarkers for relative diagnosis and therapy.

The article "Integrative Analyses of Biomarkers Associated with Endoplasmic Reticulum Stress in Ischemic Stroke" was published in 2022. Journal: Comput Math Methods Med.

## 1. Introduction

Stroke is one of the leading causes of mortality and disability worldwide. Ischemic stroke (IS) attributes to over 85% morbidity of total stroke cases [1]. Injury ensuing consequent to the interruption in cerebral blood flow, known as “ischemia and brain hypoxia,” can ultimately result in cell degeneration, apoptosis, and neurological dysfunction. Pathology of the transversion entangles a variety of cellular and biochemical molecular mechanisms, including apoptosis, neuroinflammation, oxidative stress, glutamate excitotoxicity, and energy depletion, in which neuronal apoptosis was considered to be the primary pathological metamorphosis following IS [2]. Early and effective neuroprotective therapies are needed to decrease the disability and mortality rates of IS [3]. However, the complexity of its pathophysiological mechanisms poses a major challenge to clinical treatments, and effective neuroprotectors have not been established yet [4]. Therefore, it is of great demand to explore the molecular mechanisms that regulate neuronal apoptosis and identify potential biomarkers for improvement of the current diagnostic and therapeutic procedures.

Numerous reports have confirmed that cerebral ischemia-induced ERS is a critical precipitating factor of neuronal apoptosis [5]. Endoplasmic reticulum (ER) conducts the proper folding and assembly of secretory and membranous proteins. However, when ER homeostasis is disturbed, unfolded and misfolded proteins accumulate in the ER lumen, resulting in ER stress (ERS). ERS can trigger neuronal apoptosis by multiple mechanisms, including inducing calcium overload, suppressing protein synthesis, and activating the inflammatory signal pathways [6]. Previous reports have shown that ERS may be a potential target for the diagnosis and treatment of IS; however, the key biomarkers of ERS in IS injury have not been identified yet [7]. Among all kinds of biomarkers, blood-based biomarkers contain a notable preponderance, such as minimal invasiveness, cost-effectiveness, high patient acceptability, and availability in different clinical settings [8]. The combination of microarray techniques and bioinformatics analysis was classified as a high-throughput, effective, and comprehensive method to detect the objective biomarkers [9]. Thus, we used bioinformatics analysis for the exploration of ERS blood-based biomarkers.

The aim of the present IS study is to explore the blood biomarkers associated with ERS by utilizing the whole-blood samples from the Gene Expression Omnibus (GEO) database. Differentially expressed genes (DEGs) between the patients with IS and healthy controls were identified, and the DEGs that correlated to ERS (ERS-DEGs) were further screened. Moreover, the biological functions of ERS-DEGs were analyzed via four enrichment analyses. Hub genes were screened out from ERS-DEGs via PPI analysis. Furthermore, correlation analysis and immune infiltration were used to assess the diagnostic value of the hub genes. In conclusion, the present study identified a few ERS-related biomarkers that may serve as potential determinants for further diagnosis and treatment of IS.

The article "Integrative Analyses of Biomarkers Associated with Endoplasmic Reticulum Stress in Ischemic Stroke" was published in 2022. Journal: Comput Math Methods Med.

## 2. Materials and Methods

### 2.1. Data Download and Preprocess

GEO (http://www.ncbi.nlm.nih.gov/geo) [10] is a free-accessible database that provides reliable profiles of IS, from where two gene expression profiles, GSE16561 [11] and GSE37587 [12], were searched with the keyword “ischemic stroke” and downloaded originally via GEOquery package [13] of R software V.3.6.5 (http://www.r-project.org/). Data type description is termed “expression profiling by array,” and the species is Homo sapiens. The platform for both databases is “GPL6883 Illumina HumanRef-8 v3.0 expression beadchip,” which comprises a total of 131 human whole-blood samples. Specifically, GSE16561 consists of the whole-blood samples of 39 patients with IS and 24 healthy controls, and GSE37587 contained 68 whole-blood samples of patients with IS. The raw datasets of GSE16561 and GSE37587 were combined. The sva package [14] was employed for background correction and data normalization, and the obtained result was demonstrated using the boxplot diagrams. Furthermore, diagrams of principal component analysis (PCA) were drawn using the ggplot2 package.

### 2.2. Identification of Differentially Expressed Genes

DEGs in the combined dataset were screened out via limma package [15] according to the inclusion criteria of adjusted *p* value < 0.05 and ∣log_2_FC | >0.1. Visualization of DEGs was plotted using the ggplot2 package along with volcano plot and heatmap. The list of ERS-related genes (ERSGs) was procured from the GeneCards database (https://www.genecards.org/) [16]. Venn diagram was applied to illustrate the intersection of corresponding genes, which are related to DEGs and ERS and thus, contributing to the filtrate, ERS-DEGs.

### 2.3. Gene Ontology (GO) and Kyoto Encyclopedia of Genes and Genomes (KEGG) Analysis

GO analysis is a conventional and pragmatic method for interpreting the characteristic biological functions of genes [17], including annotation of biological processes (BP), molecular functions (MF), and cellular components (CC). KEGG analysis provides all known biochemical pathways documented in a comprehensive biological database [18]. GO and KEGG pathway enrichment analyses for the ERS-DEGs were implemented via clusterProfiler package [19]. An adjusted *p* value < 0.05 would be considered statistically significant. Furthermore, we selected the GO/KEGG pathway terms with the highest enrichment degree to draw the network maps, respectively.

The article "Integrative Analyses of Biomarkers Associated with Endoplasmic Reticulum Stress in Ischemic Stroke" was published in 2022. Journal: Comput Math Methods Med.

### 2.4. Gene Set Enrichment Analysis (GSEA) and Gene Set Variation Analysis (GSVA)

To further evaluate the significant alterations in the functions and pathways of the gene expression matrix of ERS-DEGs, GSEA was performed using the clusterProfiler R package. Reference gene sets were selected as “c2.cp.kegg.v7.0.symbols.gmt.” Results with a false discovery rate (FDR) < 0.25 and adjusted *p* < 0.05 were set as the threshold for determining the significance of enrichment. Based on the results obtained from the GSEA, we explored the signal pathways of ERS-DEGs in IS via the GSVA R package [20]. Enrichment was considered significant for adjusted *p* < 0.05.

### 2.5. Protein–Protein Interaction Network Analysis and Hub Gene Identification

The protein-protein interaction (PPI) network of ERS-DEGs was constructed by the Retrieval of Interacting Genes (STRING) database (http://string-db.org) [21], which is an online tool to identify functional interactions. Furthermore, “cytoHubba,” a plugin in Cytoscape software, was employed to screen hub genes within the PPI network.

### 2.6. Network Analysis of Hub Genes

The online visual analytics platform NetworkAnalyst (https://www.networkanalyst.ca/) [22] was used to predict latent transcription factors (TFs) and miRNAs associated with the hub genes. The interaction of ERS-DEGs and potential TFs was evaluated using the obtained results of Gene Regulatory Networks (GRN) and gene-targeted record of ENCODE ChIP-seq data. The TF-miRNA coregulatory network and RegNetwork databases were used to explore the interactions between ERS-DEGs and potential miRNAs. The interaction data of ERS-DEGs and potential drugs was obtained from the DrugBank database and the analysis of protein-drug interactions in diseases, drugs, and chemicals.

### 2.7. Correlation Analysis of Hub Genes and Immune Infiltration

CIBERSORT is a tool used for deconvolution of the expression matrix of transcriptome, based on the principle of linear support vector regression. The tool can also be used to estimate the compositions and abundances of immune cells in a mixed cell population [23]. Thus, the gene expression data was uploaded to CIBERSORT, and the cut-off criteria for statistical significance was set at a *p* value less than 0.05. Consequently, the matrix data of infiltrating immune cells was obtained. The distribution of 22 types of infiltrating immune cells in each sample was presented on the heatmap plot using the heatmap R package. The correlation of 22 types of infiltrating immune cells was also visualized in the heatmaps, drawn by the corrplot package in R software.

The article "Integrative Analyses of Biomarkers Associated with Endoplasmic Reticulum Stress in Ischemic Stroke" was published in 2022. Journal: Comput Math Methods Med.

## 3. Results

### 3.1. Preprocessing of Datasets and Identification of DEGs

The two gene expression datasets (GSE16561 and GSE37587) of blood samples were first merged. The resulting single dataset was normalized and standardized prior to analysis. Illustration of datasets before and after calibration is shown in the boxplots (Figures 1(a) and 1(b)). We proceeded to evaluate the variations between healthy controls and the IS group via PCA and sample clustering analysis. As shown in Figures 1(c) and 1(d), the clustering of each group was more marked following the data preprocessing. Hence, the sample data were considered as a reliable source.

Following data preprocessing, a total of 60 DEGs; including 38 downregulated genes and 22 upregulated genes, were extracted from the gene expression matrix. This is shown in the heatmap and volcano plots (Figures 2(a) and 2(b)). Subsequently, a total of 7092 ERSGs were sorted out from the GeneCards database, and Venn diagram was applied to visualize the overlap and differences between DEGs and ERSGs. The two datasets showed an overlap of 27 ERS-DEGs (Figure 2(c)).

### 3.2. KEGG and GO Enrichment Analysis of ERS-DEGs

GO analysis results indicate that the upregulated ERS-DEGs were significantly enriched in BP pathways, including immune response-activating cell surface receptor signaling pathway, immune response-activating signal transduction, neutrophil degranulation, and neutrophil activation; all of which are involved in immune homeostasis. As for MF and CC analysis, the ERS-DEGs were mainly implicated with the external side of plasma membrane and MHC class II receptor activity, respectively (Figures 3(a)–3(d)). The results are detailed in Table 1. KEGG pathway analysis demonstrated that the upregulated ERS-DEGs were predominantly enriched in immune-related pathways, including leishmaniasis, staphylococcus aureus infection, Th17 cell differentiation, systemic lupus erythematosus, phagosome, and tuberculosis (Figures 3(e) and 3(f)). These results are shown in detail in Table 2. The pathways that were most significantly enriched from ERS-DEGs in GO and KEGG analysis are shown in diagrams (Figures 3(g) and 3(h)).

### 3.3. GSEA and GSVA

GSEA was performed to identify the biological pathways with significant alterations towards IS pathology. A total of 10 pathways were enriched by this method. Interestingly, five of them were closely associated with T cells, including T cytotoxic, T helper, IL17, NO2IL12, and CTL pathways (Figures 4(a)–4(j)). The results are detailed in Table 3. Furthermore, GSVA was conducted to further explore the signal pathways in IS, including GNF2_CD33, GSE 3688 STAT5 AB knockin vs WT T cell IL 2 T-related 17h DN, and GSE29618_monocyte_vs_PDC_up (Figure 5).

The article "Integrative Analyses of Biomarkers Associated with Endoplasmic Reticulum Stress in Ischemic Stroke" was published in 2022. Journal: Comput Math Methods Med.

### 3.4. PPI Network Analysis

To identify the interactions of the ERS-DEGs, PPI network of ERS-DEGs was established and is shown in Figure 6(a). The identified hub genes, predicted via cytoHubba plugin is also shown in the aforementioned figure. The top 10 hub genes in an increasing order of interaction degree are as follows: HIF1A, CREBBP, EP300, ARNT, TP53, PPARG, VHL, EPAS1, HIF1AN, and CREB1 (Figure 6(b)). The hub genes may be key ERS-related biomarkers of IS, which require further clinical trials for validation.

### 3.5. Network Analysis of Hub Genes

Transcriptional regulatory network analysis was performed to analyze the interaction between TFs and the hub genes (Figure 7(a)). The top 3 hub genes associated with TFs were TP53, EPAS1, and VHL. Moreover, a network of miRNAs and hub genes was constructed (Figure 7(b)). The top 3 hub genes associated with miRNAs were TP53, CREB1, and HIF1A. As potential therapeutic targets, relative drugs and molecular compounds of the hub genes were also explored by the drug-gene interaction networks. As shown in Figure 7(c), a total of 7 drugs or molecular compounds were found to interact with hub genes of HIF 1A, CREB1, and HIF1AN. They are carvedilol, 2-methoxyestradiol, N-[(1-chloro-4-hydroxyisoquinolin-3-YL)carbonyl] glycine, naloxone, adenosine monophosphate, D-tartaric acid, and N-(carboxyvarbonyl)-D-phenylalanine.

### 3.6. Immune-Related Gene Identification and Functional Correlation Analysis

The result of the CIBERSORT analysis revealed that the T and NK cell subtypes were predominant among the 22 types of infiltrating immune cells (Figure 8(a)). The correlation between 22 immune cell subtypes was also performed and presented via heatmap. The result revealed that M0 macrophages and resting NK cells had the strongest and weakest correlation with other immune cells, respectively (Figure 8(b)). Furthermore, the hub genes, ARNT, CREB1, CREBBP, EP300, EPAS1, HIF 1A, HIF 1AN, and TP53, were identified, and they correlated with 11 different types of immune cells (Figure 8(c)). We found a significant correlation between the number of neutrophil and T cell subtypes and the expression level of hub genes. The results suggested that neutrophils and T cells play a critical role in the development of ERS following IS.

The article "Integrative Analyses of Biomarkers Associated with Endoplasmic Reticulum Stress in Ischemic Stroke" was published in 2022. Journal: Comput Math Methods Med.

## 4. Discussion

IS is the primary cause of mortality and disability among Chinese residents, and its morbidity has increased over the last decade, thus, posing a huge burden to national medical and economic systems [24]. Neuronal apoptosis is the key etiological factor of neuronal damage following cerebral ischemia. Activated ERS has been reported to play a critical role in inducing neuronal cell apoptosis in IS [25]. Therefore, exploring potential biomarkers related to ERS is indispensable for the elucidation of neuronal damage following IS. However, ERS biomarkers in IS have not yet been fully identified. In this study, we comprehensively analyzed two mRNA microarray datasets (GSE16561 and GSE37587), including 107 and 24 whole-blood samples from reliable profiles of IS and healthy controls, respectively. A total of 60 DEGs were distinguished from the two datasets, including 38 and 22 downregulated and upregulated genes, respectively. Subsequently, the intersection analysis of DEGs and ERSGs was performed to obtain 27 ERS-DEGs. Enrichment analysis revealed that the modules and pathways ERS-DEGs enriched in were closely related to immunity. The data suggest that local inflammation may be involved in the development of IS. Moreover, we constructed a PPI network, and 10 hub genes with the highest scores in ERS-DEGs were identified. Our results suggested that the identified hub genes may interact with each other in the network and are also associated with immune cell infiltration.

ERS is a pathological condition related to hypoxia, starvation, calcium imbalance, and free radical excess. Contrarily, ERS can trigger the unfolded protein response, which restores homeostasis by decreasing protein translation and upregulation of ER chaperone gene expression [26]. Interestingly, unregulated ERS can initiate neuronal apoptosis by activating apoptosis signal pathways directly and also further exacerbates neuronal damage through activating inflammatory signal pathways. Recent studies have reported that ERS is a major cause of neuronal apoptosis [27]. A previous study has revealed that the promotion of ERS via knockdown Hes1 induced vast neuronal apoptosis in a mouse model with middle cerebral artery occlusion (MCAO) [25]. In addition, Li et al. reported that the inhibition of ERS signal pathway by *γ*-glutamylcysteine attenuated neuronal apoptosis in the ischemic brain of mice [28]. The aforementioned results support the idea that ERS may be a potential target in IS injury. Therefore, exploring biomarkers of ERS in blood samples of patients with IS is necessary for early diagnosis and treatment. Furthermore, it may aid the identification of novel therapeutic targets.

The article "Integrative Analyses of Biomarkers Associated with Endoplasmic Reticulum Stress in Ischemic Stroke" was published in 2022. Journal: Comput Math Methods Med.

To investigate the involvement of ERS-DEGs in the biological mechanism of IS, GO and KEGG enrichment analyses were performed, and the results revealed that ERS-DEGs are mainly enriched in immune-related pathways. In the BP annotations, neutrophil degranulation and neutrophil activation involved in immune response were found to be significantly related to the development of IS. Neutrophils are the first inflammatory responders to be recruited to the site of cerebral infarction after IS [29]. Enhanced ERS was suggested to be associated with severe neutrophil inflammation [30]. Notably, activated neutrophils release neutrophil argininase-1, which induces cell apoptosis through the ERS pathway [31]. Clinical researches have established that neutrophil overexpression is a positive indicator of stroke progression [32]. Further research has shown that inhibition of neutrophil infiltration into ischemic lesions decreases infarct size and mitigates stroke pathology [33]. These results are similar to our predictions.

Similarly, GSEA and GSVA enrichment analyses also revealed that ERS-DEGs were significantly enriched in T cell-related pathways, including T cytotoxic, T helper, IL17, NO2IL12, and CTL pathways. The results above indicate that T cells play an important role in IS. Few researchers have observed significant increases in CD4^+^ and CD8^+^ T cells in the peri-infarct area one month following IS experiments [34]. Persistent neuronal ERS has been reported to promote CD4^+^ and CD8^+^ T cell priming by inducing activation of STING signal cascade [35]. Several studies have reported that CD8^+^ T cells could induce neuronal damage directly by the cytotoxic function, while CD4^+^ T cells could aggravate the local inflammation by activating the effector T cell. Researches supported that T cell-targeted therapy could effectively reduce the infarct size of brain tissues by depleting T cells [34, 36]. In summary, our results further confirmed that T cell responses associated with ERS play an integral role in post-IS neuroinflammation.

In addition, among the 20 KEGG-enriched signaling pathways, we observed that the pathway with high enrichment was Th17 cell differentiation. In previous studies, Th17 cells were observed to be differentiated from CD4^+^ T cell in response to TGF-*β* and IL-6 and can as well produce proinflammatory cytokines. However, the unstable and plastic Th17 cells can also be transdifferentiated into Treg cells, which can attenuate inflammation [37]. Hence, T cells have a dual role in the inflammatory response after stroke. ERS was reported one of the mechanisms that deregulate Th17/Treg cells [38]. Therefore, suppressing ERS may be the effective therapeutic approach that regulated the balance between proinflammatory and anti-inflammatory mechanisms. In summary, ERS is indispensable for inflammatory responses, and our results are consistent with these findings.

The article "Integrative Analyses of Biomarkers Associated with Endoplasmic Reticulum Stress in Ischemic Stroke" was published in 2022. Journal: Comput Math Methods Med.

PPI molecular interaction network was employed to analyze the protein interaction of ERS-DEGs. Hypoxia inducible factor 1 subunit alpha (HIF1A) was identified as one of the top hub genes in this study, which is an important transcription factor in the hypoxic or ischemic brain and aids cells in the adaptation to hypoxic conditions [39]. During hypoxia, the upregulation of HIF1A can induce glycolysis and inhibit mitochondrial respiration to decrease oxygen consumption, thus, improving cell proliferation. Researches support the important role of HIF1A as a neuroprotector in ischemic brain injury [40]. Furthermore, other members in the hypoxia-inducible factor family, including EPAS1 (HIF2A) and ARNT (HIF1*β*) genes, were also identified as hub genes. Notably, cAMP response element-binding protein 1 (CREB1), was also reported as one of the hub genes that are related to neuronal survival after ischemia. CREB-related therapeutics have extensive application prospects in cerebral protection after IS [41]. Although the CREB1 inhibitor, naloxone, is conventionally used for the treatment of opioid addiction, its neurorestorative effects have been observed in patients with IS and MCAO mouse models [42]. Hence, our results indicate that the hypoxia-inducible factor family and CREB family genes are potential therapeutic targets and biomarkers of ERS in IS.

Our results indicate that CREB binding protein (CREBBP) is the top hub gene in the PPI network analysis. It has been reported to have an increased expression after IS and to be involved in neurovascular reconstruction and neuron protection [43]. Moreover, persistent ERS can promote the stability of CREBBP [44]. These findings are consistent with our results, which suggest that CREBBP may be a potential biomarker of ERS in IS. An analogue of CREBBP, EP300, was also identified as a hub gene in the PPI network. It participates in mediating the ubiquitination and degradation of CHOP protein and prevents ERS-induced apoptosis under hypoxic conditions [45]. This hub gene has been previously reported as a potential biomarker of IS, which is consistent with our report. However, the function of EP300 in IS pathology has not yet been elucidated [46]. Therefore, as a potential biomarker of IS, future investigation of EP300 is worthwhile.

In the correlation analysis between hub genes and TF or hub genes and miRNA, TP53 was found to have rich networks. Previous reports have shown that ERS can induce significant upregulation of TP53 [47]. Rapid and substantial accumulation of TP53 was observed in the ischemic penumbra, which resulted in neuronal apoptosis [48]. Therefore, TP53 may be a potential therapeutic target of IS. Interestingly, it has been reported that the inhibition of TP53 can considerably decrease infarct size [49]. Our results are consistent with the aforementioned reports, indicating that TP53 may be a potential biomarker of IS. Further investigation of the molecular mechanisms of hub genes in IS may provide novel innovations for the diagnosis and treatment of IS.

The article "Integrative Analyses of Biomarkers Associated with Endoplasmic Reticulum Stress in Ischemic Stroke" was published in 2022. Journal: Comput Math Methods Med.

However, there are several limitations to this study. First, the results were not backed up with experiments *in vitro* and *in vivo*, to further verify the biological functions of these potential ERSGs after IS. Secondly, the research was not able to evaluate the correlation between hub genes and severity of pathology in patients with IS, due to a lack of corresponding clinical studies. We also observed that the batch differences cannot be avoided and removed by the analysis, due to high-content datasets. Thus, a larger sample size and clinical study setting are required for further studies, in order to strengthen the statistical power and obtain more reliable results. Related experimental evidence is also required to fully elucidate the role of the hub genes at the molecular cellular level in IS. In addition, considering that protein biomarkers are more reliable and applicable than gene biomarkers in clinical practices, proteomics data is required for further validation of our results.

## 5. Conclusions

In conclusion, we performed a comprehensive analysis of the differentially expressed genes associated with ERS following IS, by combining two datasets (GSE16561 and GSE37587) to explore the molecular mechanism and biomarkers of ERS, which are involved in neuronal damage of IS. ERS-DEGs and hub genes were identified, which may be potential therapeutic targets and biomarkers of IS. Enrichment analysis indicated that the immune-related signal pathway is an assignable mechanism in the progression of IS. Network and immune correlation analyses further confirmed that the identified hub genes are closely related to immune infiltration. However, further clinical studies should be conducted in order to validate our findings.

## Figures and Tables

**Figure 1:** Illustration of GSE16561 and GSE37587 datasets before and after calibration. (a, b) The boxplot diagrams of the datasets with the interbatch difference were removed before and after to calibration. (c, d) The PCA diagrams of the datasets with the interbatch difference were removed before and after calibration.

The article "Integrative Analyses of Biomarkers Associated with Endoplasmic Reticulum Stress in Ischemic Stroke" was published in 2022. Journal: Comput Math Methods Med.

**Figure 2:** ERS-DEGs were obtained from the intersection of DEGs and ERS-related genes. (a) Heatmap of DEGs; (b) volcano plot of the distributions of DEGs. Red and blue dots represent upregulated and downregulated genes, respectively. No significantly changed genes were marked as grey dots; (c) Venn diagram of ERS-DEGs. Venn diagram analysis executed an intersection of DEGs and ERSGs to reveal the ERS-DEGs.

**Figure 3:** GO/KEGG enrichment analyses of ERS-DEGs. (a) Advanced bubble chart shows GO functional enrichment significance items of ERS-DEGs in three functional groups: BP, MF, and CC. The *x*-axis and *y*-axis labels represent the gene ratios enriched in the GO analysis group and GO terms, respectively. The color of dots represents the adjusted *p* value: the redder the color, the lesser the adj. *p* value; the bluer the color, the greater the adj. *p* value. The size of dots represents gene counts. (b–d) Chord diagrams show the distribution of ERS-DEGs in the three different GO-enriched functions. The color of dots represents the log FC of the genes. (e) Advanced bubble chart shows enrichment of ERS-DEGs in signal pathways. (f) The chord diagram shows the distribution of ERS-DEGs in different KEGG pathways. (g) The pathway diagram shows the immune response-activating cell surface receptor signaling pathway with the highest enrichment degree in GO analysis. (h) The pathway diagram shows that the leishmaniasis pathway has the highest enrichment degree in KEGG analysis.

**Figure 4:** The top 10 significantly enriched pathways based on GSEA. (a) WP purine metabolism; (b) BioCarta T cytotoxic pathway; (c) BioCarta T helper pathway; (d) Reactome mRNA decay by 3′ to 5′ exoribonuclease; (e) BioCarta IL17 pathway; (f) Reactome transport of nucleoside-free purine and pyrimidine bases across the plasma membrane; (g) KEGG primary immunodeficiency; (h) BioCarta NO2IL12 pathway; (i) BioCarta CTL pathway; (j) Reactome mitochondrial calcium ion transport.

**Figure 5:** Heatmap of 10 signal pathways of ERS-DEGs based on GSVA.

**Figure 6:** Protein–protein interaction (PPI) networks. (a) PPI network analysis of ERS-DEGs. Red and blue colors represent high and low expression levels of genes, respectively. (b) The top 10 hub genes from the PPI network were predicted and shown on the subnetwork. Node color reflects the degree of accuracy in prediction with a gradient shift from yellow to red. Illustratively, the redder the color, the higher the accuracy of prediction.

**Figure 7:** Network analyses of the hub genes. (a) Network of hub gene-TFs. Dots in blue to green represent the hub genes, and dots in red to yellow represent the TFs. (b) Network of hub gene-miRNA. Red and blue nodes are hub genes and miRNAs, respectively. (c) Networks of hub gene-related drug. Red and blue circle nodes are hub genes and drugs/molecular compounds, respectively.

The article "Integrative Analyses of Biomarkers Associated with Endoplasmic Reticulum Stress in Ischemic Stroke" was published in 2022. Journal: Comput Math Methods Med.

**Figure 8:** The nose cone is detachable upon impact. Evaluation and visualization of infiltrating immune cells. (a) Bar diagram displayed the proportion of infiltrating immune cells based on CIBERSORT algorithm. (b) Heatmap of the correlation between 22 subtypes of immune cells. Blue and red areas indicate positive and negative correlations, respectively. The darker the color, the stronger the correlation. (c) The correlations between hub genes and immune cells.

**Table 1:** GO enrichment analysis of ERS-DEGs.

Ontology	ID	Description	GeneRatio	BgRatio	*p* value	*p*.adjust	*q* value
BP	GO:0043312	Neutrophil degranulation	12/49	485/18670	3.18*e*-09	1.67*e*-06	1.30*e*-06
BP	GO:0002283	Neutrophil activation involved in immune response	12/49	488/18670	3.41*e*-09	1.67*e*-06	1.30*e*-06
BP	GO:0042119	Neutrophil activation	12/49	498/18670	4.28*e*-09	1.67*e*-06	1.30*e*-06
BP	GO:0002446	Neutrophil mediated immunity	12/49	499/18670	4.38*e*-09	1.67*e*-06	1.30*e*-06
BP	GO:0030098	Lymphocyte differentiation	9/49	353/18670	2.94*e*-07	8.99*e*-05	7.00*e*-05
CC	GO:0009897	External side of plasma membrane	11/50	393/19717	3.19*e*-09	4.09*e*-07	2.76*e*-07
CC	GO:0042581	Specific granule	7/50	160/19717	1.51*e*-07	9.69*e*-06	6.53*e*-06
CC	GO:0070820	Tertiary granule	6/50	164/19717	3.55*e*-06	1.51*e*-04	1.02*e*-04
CC	GO:1904724	Tertiary granule lumen	4/50	55/19717	1.13*e*-05	3.54*e*-04	2.38*e*-04
CC	GO:0034774	Secretory granule lumen	7/50	321/19717	1.56*e*-05	3.54*e*-04	2.38=-04
MF	GO:0019864	IgG binding	2/49	11/17697	4.07*e*-04	0.073	0.058

**Table 2:** KEGG enrichment analysis of ERS-DEGs.

Ontology	ID	Description	GeneRatio	BgRatio	*p* value	*p*.adjust	*q* value
KEGG	hsa04640	Hematopoietic cell lineage	5/32	99/8076	3.87*e*-05	0.004	0.004
KEGG	hsa05140	Leishmaniasis	4/32	77/8076	2.24*e*-04	0.013	0.010
KEGG	hsa05340	Primary immunodeficiency	3/32	38/8076	4.34*e*-04	0.015	0.012
KEGG	hsa05150	Staphylococcus aureus infection	4/32	96/8076	5.22*e*-04	0.015	0.012
KEGG	hsa04659	Th17 cell differentiation	4/32	107/8076	7.87*e*-04	0.018	0.014

**Table 3:** GSEA in IS.

ID	Description	Set size	Enrichment score	NES	*p* value	*p*.adjust	*q* values	Rank
GO:0031982	Vesicle	485	0.172714697	3.411234438	0.001432665	0.004133545	0.001924525	700
GO:0005576	Extracellular region	410	0.174994196	3.266701279	0.001449275	0.004133545	0.001924525	435
GO:0005739	Mitochondrion	243	0.142281361	2.213093251	0.001464129	0.004133545	0.001924525	983
GO:0005615	Extracellular space	329	0.19021029	3.274198836	0.001474926	0.004133545	0.001924525	252
GO:0043230	Extracellular organelle	263	0.22061393	3.541020551	0.001477105	0.004133545	0.001924525	621
GO:0070062	Extracellular exosome	261	0.220698869	3.524995246	0.001477105	0.004133545	0.001924525	621
GO:1903561	Extracellular vesicle	263	0.22061393	3.541020551	0.001477105	0.004133545	0.001924525	621
GO:0030054	Cell junction	201	0.16579481	2.408482794	0.001481481	0.004133545	0.001924525	189
GO:0031410	Cytoplasmic vesicle	322	0.145729015	2.48768047	0.001481481	0.004133545	0.001924525	589
GO:0097708	Intracellular vesicle	322	0.145729015	2.48768047	0.001481481	0.004133545	0.001924525	589
GO:0031967	Organelle envelope	204	0.186841967	2.730329262	0.001485884	0.004133545	0.001924525	788
GO:0031975	Envelope	204	0.186841967	2.730329262	0.001485884	0.004133545	0.001924525	788
GO:0030141	Secretory granule	150	0.225718868	2.855414686	0.001497006	0.004133545	0.001924525	404
GO:0098796	Membrane protein complex	150	0.162131482	2.051014249	0.001497006	0.004133545	0.001924525	656
GO:0099503	Secretory vesicle	171	0.222023193	2.994872073	0.001510574	0.004133545	0.001924525	404
GO:0005740	Mitochondrial envelope	137	0.190035312	2.306946726	0.001529052	0.004133545	0.001924525	616
GO:1990904	Ribonucleoprotein complex	129	0.179654365	2.131343914	0.001531394	0.004133545	0.001924525	902
GO:0031966	Mitochondrial membrane	130	0.177934672	2.116907669	0.001533742	0.004133545	0.001924525	616
GO:0019866	Organelle inner membrane	100	0.24461389	2.624119415	0.001572327	0.004133545	0.001924525	609
GO:0070161	Anchoring junction	104	0.251547714	2.735235303	0.001589825	0.004133545	0.001924525	149
GO:0012506	Vesicle membrane	121	0.174348266	1.997474797	0.00311042	0.007397923	0.003444377	1110
GO:0030659	Cytoplasmic vesicle membrane	118	0.177306426	2.00809075	0.00312989	0.007397923	0.003444377	1110
GO:0031090	Organelle membrane	474	0.102433696	2.016629844	0.004341534	0.009815642	0.004570036	656
GO:0000228	Nuclear chromosome	129	-0.149453948	-1.990943144	0.005730659	0.012416428	0.005780928	647
GO:1902494	Catalytic complex	204	0.125116027	1.828325596	0.013372957	0.02781575	0.012950653	1192
GO:0045202	Synapse	122	0.147449379	1.693366467	0.020344288	0.040688576	0.018944074	167
GO:0000790	Nuclear chromatin	107	-0.137337172	-1.666983644	0.024456522	0.047101449	0.021929825	621

The article "Integrative Analyses of Biomarkers Associated with Endoplasmic Reticulum Stress in Ischemic Stroke" was published in 2022. Journal: Comput Math Methods Med.

## Data Availability

The datasets used and/or analyzed during the current study are available from the corresponding authors on reasonable request.

## References

[1] Jayaraj R. L., Azimullah S., Beiram R., Jalal F. Y., Rosenberg G. A. (2019). Neuroinflammation: friend and foe for ischemic stroke. *Journal of Neuroinflammation*.

[2] Liu R., Tang J. C., Pan M. X. (2018). ERK 1/2 Activation Mediates the Neuroprotective Effect of BpV(pic) in Focal Cerebral Ischemia–Reperfusion Injury. *Neurochemical Research*.

[3] Kam K. Y., Yu S. J., Jeong N. (2011). p-Hydroxybenzyl alcohol prevents brain injury and behavioral impairment by activating Nrf2, PDI, and neurotrophic factor genes in a rat model of brain ischemia. *Molecules and Cells*.

[4] Li Y., Xiang L. L., Miao J. X., Miao M. S., Wang C. (2021). Protective effects of andrographolide against cerebral ischemia‑reperfusion injury in mice. *International Journal of Molecular Medicine*.

[5] Han Y., Yuan M., Guo Y. S., Shen X. Y., Gao Z. K., Bi X. (2021). Mechanism of endoplasmic reticulum stress in cerebral ischemia. *Frontiers in Cellular Neuroscience*.

[6] Ghosh R., Wang L., Wang E. S. (2014). Allosteric inhibition of the IRE1*α* RNase preserves cell viability and function during endoplasmic reticulum stress. *Cell*.

[7] Liu S., Xin D., Wang L. (2017). Therapeutic effects of L-Cysteine in newborn mice subjected to hypoxia-ischemia brain injury via the CBS/H_2_S system: Role of oxidative stress and endoplasmic reticulum stress. *Redox Biology*.

[8] Mielke M. M., Syrjanen J. A., Blennow K. (2019). Plasma and CSF neurofilament light: relation to longitudinal neuroimaging and cognitive measures. *Neurology*.

[9] Li Z., Cui Y., Feng J., Guo Y. (2020). Identifying the pattern of immune related cells and genes in the peripheral blood of ischemic stroke. *Journal of Translational Medicine*.

[10] Barrett T., Wilhite S. E., Ledoux P. (2013). NCBI GEO: archive for functional genomics data sets—update. *Nucleic Acids Research*.

[11] Barr T. L., Conley Y., Ding J. (2010). Genomic biomarkers and cellular pathways of ischemic stroke by RNA gene expression profiling. *Neurology*.

[12] Barr T. L., Van Gilder R., Rellick S. (2015). A genomic profile of the immune response to stroke with implications for stroke recovery. *Biological Research for Nursing*.

[13] Davis S., Meltzer P. S. (2007). GEOquery: a bridge between the Gene Expression Omnibus (GEO) and BioConductor. *Bioinformatics*.

[14] Leek J. T., Johnson W. E., Parker H. S., Jaffe A. E., Storey J. D. (2012). The sva package for removing batch effects and other unwanted variation in high-throughput experiments. *Bioinformatics*.

[15] Ritchie M. E., Phipson B., Wu D. (2015). limma powers differential expression analyses for RNA-sequencing and microarray studies. *Nucleic Acids Research*.

[16] Stelzer G., Rosen N., Plaschkes I. (2016). The GeneCards suite: from gene data mining to disease genome sequence analyses. *Current Protocols In Bioinformatics*.

[17] Ashburner M., Ball C. A., Blake J. A. (2000). Gene ontology: tool for the unification of biology. *Nature Genetics*.

The article "Integrative Analyses of Biomarkers Associated with Endoplasmic Reticulum Stress in Ischemic Stroke" was published in 2022. Journal: Comput Math Methods Med.

[18] Ogata H., Goto S., Sato K., Fujibuchi W., Bono H., Kanehisa M. (1999). KEGG: Kyoto Encyclopedia of Genes and Genomes. *Nucleic Acids Research*.

[19] Yu G., Wang L. G., Han Y., He Q. Y. (2012). clusterProfiler: an R package for comparing biological themes among gene clusters. *OMICS: A Journal of Integrative Biology*.

[20] Hanzelmann S., Castelo R., Guinney J. (2013). GSVA: gene set variation analysis for microarray and RNA-seq data. *BMC Bioinformatics*.

[21] Szklarczyk D., Gable A. L., Lyon D. (2019). STRING v11: protein–protein association networks with increased coverage, supporting functional discovery in genome-wide experimental datasets. *Nucleic Acids Research*.

[22] Zhou G., Soufan O., Ewald J., Hancock R. E. W., Basu N., Xia J. (2019). NetworkAnalyst 3.0: a visual analytics platform for comprehensive gene expression profiling and meta-analysis. *Nucleic Acids Research*.

[23] Newman A. M., Liu C. L., Green M. R. (2015). Robust enumeration of cell subsets from tissue expression profiles. *Nature Methods*.

[24] Zhang X., Zhou G. (2020). MiR-199a-5p inhibition protects cognitive function of ischemic stroke rats by AKT signaling pathway. *American Journal of Translational Research*.

[25] Li Y., Zhang Y., Fu H. (2020). Hes1 knockdown exacerbates ischemic stroke following tMCAO by increasing ER stress-dependent apoptosis via the PERK/eIF2*α*/ATF4/CHOP signaling pathway. *Neuroscience Bulletin*.

[26] Pan B., Sun J., Liu Z. (2021). Longxuetongluo Capsule protects against cerebral ischemia/reperfusion injury through endoplasmic reticulum stress and MAPK-mediated mechanisms. *Journal of Advanced Research*.

[27] Cao G., Zhou H., Jiang N. (2016). YiQiFuMai powder injection ameliorates cerebral ischemia by inhibiting endoplasmic reticulum stress-mediated neuronal apoptosis. *Oxidative Medicine and Cellular Longevity*.

[28] Li H. Q., Xia S. N., Xu S. Y. (2021). *γ*-Glutamylcysteine alleviates ischemic stroke-induced neuronal apoptosis by inhibiting ROS-mediated endoplasmic reticulum stress. *Oxidative Medicine and Cellular Longevity*.

[29] Chu H. X., Kim H. A., Lee S. (2014). Immune cell infiltration in malignant middle cerebral artery infarction: comparison with transient cerebral ischemia. *Journal of Cerebral Blood Flow & Metabolism*.

[30] Pathinayake P. S., Waters D. W., Nichol K. S. (2022). Endoplasmic reticulum-unfolded protein response signalling is altered in severe eosinophilic and neutrophilic asthma. *Thorax*.

[31] Garcia-Navas R., Gajate C., Mollinedo F. (2021). Neutrophils drive endoplasmic reticulum stress-mediated apoptosis in cancer cells through arginase-1 release. *Scientific Reports*.

The article "Integrative Analyses of Biomarkers Associated with Endoplasmic Reticulum Stress in Ischemic Stroke" was published in 2022. Journal: Comput Math Methods Med.

[32] Maestrini I., Strbian D., Gautier S. (2015). Higher neutrophil counts before thrombolysis for cerebral ischemia predict worse outcomes. *Neurology*.

[33] Jickling G. C., Liu D., Ander B. P., Stamova B., Zhan X., Sharp F. R. (2015). Targeting neutrophils in ischemic stroke: translational insights from experimental studies. *Journal of Cerebral Blood Flow & Metabolism*.

[34] Lei T. Y., Ye Y. Z., Zhu X. Q. (2021). The immune response of T cells and therapeutic targets related to regulating the levels of T helper cells after ischaemic stroke. *Journal of Neuroinflammation*.

[35] Sen T., Saha P., Gupta R. (2020). Aberrant ER stress induced neuronal-IFN*β* elicits white matter injury due to microglial activation and T-cell infiltration after TBI. *Journal of Neuroscience*.

[36] Liesz A., Zhou W., Mracsko E. (2011). Inhibition of lymphocyte trafficking shields the brain against deleterious neuroinflammation after stroke. *Brain*.

[37] Gagliani N., Amezcua Vesely M. C., Iseppon A. (2015). Th17 cells transdifferentiate into regulatory T cells during resolution of inflammation. *Nature*.

[38] Xiao D., Li S., Gui B. (2020). Effect of uremic serum on Th17/Treg cell balance and endoplasmic reticulum stress in rats. *Biomedicine & Pharmacotherapy*.

[39] Yang J., Liu C., Du X. (2018). Hypoxia inducible factor 1*α* plays a key role in remote ischemic preconditioning against stroke by modulating inflammatory responses in rats. *Journal of the American Heart Association*.

[40] Ogle M. E., Gu X., Espinera A. R., Wei L. (2012). Inhibition of prolyl hydroxylases by dimethyloxaloylglycine after stroke reduces ischemic brain injury and requires hypoxia inducible factor-1*α*. *Neurobiology of Disease*.

[41] Kitagawa K. (2007). CREB and cAMP response element-mediated gene expression in the ischemic brain. *The FEBS Journal*.

[42] Peyravian N., Dikici E., Deo S., Toborek M., Daunert S. (2019). Opioid antagonists as potential therapeutics for ischemic stroke. *Progress in Neurobiology*.

[43] Zhu X., Liu X., Liu Y., Chang W., Song Y., Zhu S. (2020). Uncovering the potential differentially expressed miRNAs and mRNAs in ischemic stroke based on integrated analysis in the gene expression omnibus database. *European Neurology*.

[44] Liu B., Zhang Z., Hu Y. (2019). Sustained ER stress promotes hyperglycemia by increasing glucagon action through the deubiquitinating enzyme USP14. *Proceedings of the National Academy of Sciences*.

[45] Jeong K., Kim H., Kim K. (2014). Cyclophilin B is involved in p300-mediated degradation of CHOP in tumor cell adaptation to hypoxia. *Cell Death & Differentiation*.

The article "Integrative Analyses of Biomarkers Associated with Endoplasmic Reticulum Stress in Ischemic Stroke" was published in 2022. Journal: Comput Math Methods Med.

[46] Wang Y., Feng F., Zheng P. (2022). Dysregulated lncRNA and mRNA may promote the progression of ischemic stroke via immune and inflammatory pathways: results from RNA sequencing and bioinformatics analysis. *Genes & Genomics*.

[47] Swiatkowska A., Dutkiewicz M., Machtel P. (2020). Regulation of the p53 expression profile by hnRNP K under stress conditions. *RNA Biology*.

[48] Almeida A., Sanchez-Moran I., Rodriguez C. (2021). Mitochondrial–nuclear p53 trafficking controls neuronal susceptibility in stroke. *IUBMB Life*.

[49] Lu J., Xu F., Lu H. (2020). LncRNA PVT1 regulates ferroptosis through miR-214-mediated TFR1 and p53. *Life Sciences*.

